RETRACTED

# Cell Surface GRP78 Accelerated Breast Cancer Cell Proliferation and Migration by Activating STAT3

**DOI:** 10.1371/journal.pone.0125634

**Published:** 2015-05-14

**Authors:** Xiaoli Yao, Hua Liu, Xinghua Zhang, Liang Zhang, Xiang Li, Changhua Wang, Shengrong Sun

**Affiliations:** 1 Department of Breast and Thyroid Surgery, Renmin Hospital of Wuhan University, Wuhan, 430060, Hubei Province, China; 2 Department of Clinical Pathology, The First People’s Hospital of Lianyungang, Lianyungang, 222000, Jiangsu Province, China; 3 Department of Pathophysiology, Wuhan University School of Basic Medical Sciences, Wuhan, 430071, Hubei Province, China; 4 Department of Urology, Renmin Hospital of Wuhan University, Wuhan, 430060, Hubei Province, China; Duke University Medical Center, UNITED STATES

## Abstract

High levels of cell surface glucose regulated protein 78 (sGRP78) have been implicated in cancer growth, survival, metastasis, and chemotherapy resistance. However, the underlying mechanism remains largely unknown. Here we report that the level of sGRP78 expression in human breast tumors gradually increases during cancer progression. Overexpression of GRP78 significantly enhanced its membrane distribution in human MCF-7 breast cancer cells, but had no effect on endoplasmic reticulum (ER) stress. High levels of sGRP78 facilitated cell proliferation and migration, as well as suppressed cell apoptosis. Neutralization of sGRP78 by a specific antibody against GRP78 alleviated sGRP78-induced cell growth and migration. Importantly, high phosphorylation levels of the signal transducer and activator of transcription 3 (STAT3) were found in human breast tumors that express sGRP78 and MCF-7 cells infected with adenovirus encoding human GRP78. Pretreatment with a GRP78 antibody suppressed STAT3 phosphorylation. Furthermore, genetic and pharmacological inhibition of STAT3 reversed the impacts of GRP78 on cell proliferation, apoptosis, and migration. These findings indicate that STAT3 mediates sGRP78-promoted breast cancer cell growth and migration.

## Introduction

Glucose regulated protein 78 (GRP78, also known as binding immunoglobulin protein (BiP)) is a multi-functional protein predominantly expressed in the lumen of the endoplasmic reticulum (ER). Typically, GRP78 acts as a major ER chaperone and a master regulator of ER stress signaling through controlling protein folding and assembly, preventing protein aggregation, and regulating signaling of the unfolded protein response (UPR) [1–4]. As a central stress sensor, the level of GRP78 can be up-regulated by a variety of alterations in the tumor microenvironment, such as hypoxia, glucose or nutrient deprivation, lactic acidosis, and inflammatory response [5]. High levels of GRP78 promote cancer cell proliferation, survival, apoptosis resistance, immune escape, metastasis, angiogenesis in the microenvironment, and resistance to therapies [6, 7]. Thus, GRP78 expression may serve as a biomarker for tumor behavior and treatment response, as well as a potential target for new therapies [6].

RETRACTED

Currently, GRP78 was found to translocate to the surface of many types of cancer cells acting as an important regulator of oncogenic signaling, cancer survival, and metastasis [5, 8–10]. Particularly, the up-regulation of cell surface GRP78 (sGRP78), both at the RNA and protein level, presents in the cell membrane of malignant cells, but not in those of benign cells [8, 11]. High levels of sGRP78 promote cancer cell proliferation, migration, apoptosis resistance, and invasion [12–14]. In contrast, neutralization of sGRP78 by a specific antibody against GRP78 suppresses tumor growth and metastasis both *in vitro* and *in vivo* [10, 15, 16].

Signal transducer and activator of transcription 3 (STAT3) plays a vital role in cell survival and tumorigenesis [17, 18]. STAT3 has been found to be constitutively activated in many cancers. Suppression of STAT3 by pharmacological agents and genetic interference inhibits cell proliferation, induces apoptosis, and suppresses tumorigenicity *in vivo* [17, 18]. Thus, STAT3 may also be considered as a prognostic marker and therapeutic target in human breast cancer [19].

In the present study, we found that sGRP78 was highly expressed in breast tumors, accompanied by the elevated STAT3 phosphorylation. Overexpression of GRP78 increased membrane distribution of GRP78 and enhanced STAT3 phosphorylation. Inhibition of sGRP78 function by a specific anti-GRP78 antibody mitigated GRP78-induced STAT3 phosphorylation. Genetic and pharmacological inhibition of STAT3 abolished sGRP78-promoted breast cancer cell growth and migration. Our results, for the first time, suggest that sGRP78-induced tumor promotion is mediated by STAT3.

## Materials and Methods

### Material and reagents

Antibodies used in this study include the following: GRP78 antibody (N-20 and C-20, Santa Cruz Biotechnology, Santa Cruz, CA, USA), Phosphos-IRE1α (Ser724) antibody (Abcam, Cambridge, UK); E-cadherin (Stressgen, Victoria, Canada); STAT3, Phospho-STAT3 (Tyr705), JAK2, Phospho-JAK2 (Tyr1007/1008), CHOP, Caspase-3, IRE1α, and PARP antibody (Cell Signaling Technology, Beverley, MD, USA); and β-tubulin antibody (Sigma-Aldrich, Steinheim, Germany). Tunicamycin was from Sigma-Aldrich. Dulbecco’s Modified Eagles Medium (DMEM), fetal bovine serum (FBS), and Geneticin (G418) were purchased from HyClone (Logan, UT, USA). STAT3 specific inhibitor benzoic acid (2-Hydroxy-4-(((4-methylphenyl)sulfonyloxy)acetyl)amino)-benzoic acid, NSC74859), human STAT3/shRNA, and control shRNA lentiviral particles were obtained from Santa Cruz Biotechnology.

RETRACTED

### Clinical Specimen and cell culture

The frozen breast tumor tissues and their paired adjacent non-tumor tissues were obtained from the Department of Clinic Pathology of Wuhan University Renmin Hospital. Written informed consent from the patients was obtained, and this series of studies was reviewed and approved by Institutional Ethics Committees of Wuhan University Renmin Hospital.

Human MCF-7 and MDA-MB-453 breast cancer cells (ATCC, Manassas, VA, USA) were cultured in DMEM supplemented with 10% FBS and 1% penicillin/streptomycin at 37°C in a humidified atmosphere containing 5% CO_2_.

### Cell proliferation assay

Cell proliferation was assessed in 96-well dishes using an 3-(4,5-dimethylthiazol-2-yl)-2,5-diphenyltetrazolium bromide (MTT) assay as described previously [20]. Briefly, 3×10^3^ cells/well were seeded in 100 μl of complete DMEM with 20% FBS. After treatment with or without the indicated compounds for certain time, the medium was removed from each well, and then 150 μl of fresh medium (without phenol red) with 50 μl of 0.5 mg/ml MTT solution was added. After incubation for 3 h at 37°C, the medium was carefully removed and 150 μl of MTT solvent was added into well. The plate was covered with tinfoil and agitated on an orbital shaker for 15 min. An ELISA plate reader (Biotek, Winooski, VT, USA) was used to determine absorbance at 590 nm with a reference filter of 620 nm.

### Apoptosis assay

The cells were incubated in serum-free medium with or without 25 ng/ml of tumor necrosis factor-alpha (TNFα) for 24 h, fixed with 3.8% paraformaldehyde for 20 min, and then stained with the terminal deoxyribonucleotidyl transferase (TdT)-mediated dUTP-digoxigenin nick end labeling (TUNEL) reagent (Roche, Basel, Switzerland) for in situ apoptosis detection. Positive and negative controls were pretreated with 10 U/ml DNase or incubated without TdT, respectively. Apoptotic cells were detected under an Olympus FluoView FV1000 Confocal Microscope.

### Wound migration assay

The cells were seeded into 6-well plates and cultured to 100% confluence. A pipette tip was used to make a straight scratch in the cell layer to create the wound. Then, the cells were washed with PBS, and treated with or without the indicated compounds. Mitomycin C (Sigma-Aldrich) was used to inhibit cell proliferation. Wound images were taken with a digital camera mounted on light microscope. The wound gap widths were measured using Image J software.

RETRACTED

### Adenovirus construction and virus infection

The construction of recombinant adenoviral vectors expressing human GRP78 (Ad/GRP78) were performed as previously described [21, 22]. A recombinant adenoviral plasmid expressing β-galactosidase (Ad/β-gal) was kindly provided by Dr. Xuejun Wang (The University of South Dakota Sanford School of Medicine, Vermillion, SD). Adenoviruses were amplified in HEK293 cells and purified with a cesium chloride gradient. MCF-7 and MDA-MB-453 cells were infected with Ad/GRP78 or a control Ad/β-gal (MOI:100,) in serum-free medium for 6 h, and then cultured in growth medium for 24 h. Lentivirus carrying human STAT3/shRNA was used to silence STAT3. Lentivirus transduction was performed according to the manufacturer's protocol.

### Membrane fraction preparation and western blot

The cells and minced tissues were sonicated in ice cold lysis buffer (containing 50 mM Hepes, pH7.6, 150 mM NaCl, 1% Triton X-100, 1 mM NaF, 20 mM sodium pyrophosphate, 20 mM β-glycerol phosphate, 1 mM sodium orthovanadate, 10 μg/ml leupeptin, 10 μg/ml aprotinin, 1 μM microcystin-LR, and 1mM phenylmethylsulfonyl fluoride) and put on ice for 10 or 20 min, respectively, and then centrifuged at 14,000 g for 10 min at 4°C. The supernatants were collected and protein concentrations were determined using a bicinchoninic acid (BCA) assay. The membrane fraction from the tissues and cells were prepared using a membrane, cytosolic and nuclear compartment protein extraction kit (Biochain Institute Inc., Hayward, CA) according to the manufacturer’s instructions. Purity of membrane fraction was determined by expression of membrane marker E-cadherin and ER maker calnexin. The proteins were separated by sodium dodecyl sulfate polyacrylamide gel electrophoresis (SDS-PAGE), transferred to a nitrocellulose membrane, and detected with specific antibodies. β-tubulin and E-cadherin served as the inner references of the cytosolic and membrane protein, respectively, for all western blots. The intensity of protein bands was quantified using Bio-Rad Quantity One software.

### Immunofluorescence

The immunofluorescence labeling of formalin-fixed paraffin-embedded (FFPE) breast cancer tissues was performed as previously described [23]. Briefly, four-micron FFPE sections were heat-treated under pressure in a microwave for 5 min, and then incubated with primary antibodies for 1 h at room temperature. Next, the sections were incubated with secondary antibodies with fluorescent labels for 1 h at room temperature. The nuclei were stained with the DNA dye DAPI. The results were randomly evaluated independently by two specialized cancer-pathologists who were masked to all clinical data. The immunofluorescence results were analyzed with the Automated Quantitative Analysis (AQUA) system.

RETRACTED

For staining of cultured cells, the cells were fixed with 3.7% paraformaldehyde, washed three times with PBS, and blocked with 1% bovine serum albumin (BSA, in PBS) for 1 h. After washing 3 times with PBS, the cells were incubated with primary antibody for 1 h at room temperature followed by washing 3 times with PBS and incubation with a second antibody conjugated to fluorescent dyes for 1 h at room temperature. Finally, the mixture was mounted with mounting solution after three additional washes. Confocal images were taken by always using the same fixed scan parameters and fixed settings.

### Statistical analysis

All values are represented as the mean ± SEM. Differences between mean values were examined using the paired Student’s *t*-test. Chi Square was used to test differences between two or more actual samples. *p*<0.05 was regarded as statistically significant. Linear regression was calculated using Pearson’s correlation analysis. The quantification of the relative increase in protein expression and phosphorylation statuses was normalized with control protein expression in each experiment. The figures are representative of at least three independent experiments with similar results.

## Results

### Cell surface GRP78 is upregulated in human breast carcinoma

We firstly analyzed a series of paired human breast tumors and adjacent non-tumor tissues for the expression pattern of cell surface GRP78 (sGRP78) by immunofluorescence (IF). sGRP78 location was determined by co-localization with the membrane marker protein E-cadherin. The level of sGRP78 was assessed according to fluorescence intensity. Representative IF sections showed that sGRP78 expression was gradually elevated with pathological tumor stage progression (Fig 1A). Western blot results (Fig 1B) also revealed that sGRP78 is highly expressed in tumors when compared with a group of matched non-tumor counterparts, suggesting a positive correlation of sGRP78 with tumorigenesis. By scoring 69 non-tumor tissues and 104 tumor tissues, we found that sGRP78 was highly stained in 17.4% of non-tumor tissues and in 65.4% of tumor tissues (p<0.01) (Fig 1C). We next investigated the correlation of sGRP78 with the clinic pathological parameters of these tumors and found that GRP78 is highly expressed in a group of tumors with a high pathological stage (Fig 1D). In addition, sGRP78 levels were positively associated with tumor size, the number of positive lymph node, grade, and pathological stage of breast cancer (Table 1). No relationship was observed between the sGRP78 expression and other characteristics such as age, menopause status, ER/PR expression, as well as Her2 expression (Table 1). Thus, our results indicated that sGRP78 expression progressively increased during cancer progression.

RETRACTED

**Fig 1:** Association of sGRP78 expression with breast tumor progression. (A) Representative immunofluorescence staining of cell surface GRP78 (sGRP78) protein in sGRP78 positive human breast carcinomas. (B) Western blotting of sGRP78 protein in breast tumor and non-tumor tissues. The expression level of sGRP78 was normalized to E-cadherin and is represented in the bottom panel. (C) The percentage of sGRP78 highly stained cases in 104 tumor tissues and 69 non-tumor tissues detected by immunofluorescence analysis. (D) Distribution of sGRP78 highly stained cases with tumor characteristics. *p<0.05, **p<0.01, ***p<0.001 vs the non-tumor group. N: non-tumor tissue; T: tumor tissue.

**Table 1:** Association between sGRP78 expression and patient clinical/pathological characteristics.

		Total	sGRP78 positive Number	p-value
**Age**	<40	16	11	
	40-<50	35	22	
	50-<60	32	20	
	>60	21	15	0.89
**Menopause**	Pre	66	47	
	Post	38	21	0.10
**Tumor size**	≤2cm	35	16	
	>2cm≤5cm	55	40	
	>5cm	14	12	0.007
**No. of positive lymph nodes**	0	34	16	
	1–3	40	28	
	4–9	18	14	
	>10	12	10	0.04
**Grade**	1	9	4	
	2	35	19	
	3	60	45	0.047
**Pathological stage**	I	29	12	
	II	41	27	
	III	34	29	0.001
**Histology**	Infiltrating ductal	92	62	
	other	12	6	0.23
**ER/PR**	-/- (-/+)or(+/+)or(+/-)	35	26	
		69	42	0.17
**Her2**	Negative	73	47	
	Positive	31	21	0.74

P-values are based on chi-square test

### Cell surface GRP78 is up-regulated in MCF-7 cells infected with Ad/GRP78

To observe the potential impact of GRP78 overexpression on its membrane distribution, GRP78 was overexpressed in MCF-7 cells which have the lowest endogenous levels of GRP78 protein [24], by infection with adenovirus encoding human GRP78 (Ad/GRP78). Adenovirus expressing β-galactosidase (Ad/β-gal) served as the control. GRP78 expression was detected by immunofluorescence staining and western blotting, respectively. In non-permeabilized cells, staining primarily detects sGRP78, rather than intracellular GRP78. As shown in Fig 2A, the immunofluorescence intensity of sGRP78 was dramatically increased in the Ad/GRP78-infected MCF-7 cells when compared to the Ad/β-gal-infected cells. This result was further confirmed by western blot showing high GRP78 expression in the membrane fraction of the Ad/GRP78-infected MCF-7 cells (Fig 2B) or MDA-MB-453 cells (S1 Fig). When sGRP78 expression was normalized with the membrane marker protein E-cadherin, Ad/GRP78-infection drove a 2.9-fold increase in sGRP78 when compared with Ad/β-gal-infected MCF-7 cells (Fig 2C).

RETRACTED

**Fig 2:** Overexpression of GRP78 in MCF-7 cells. (A) Cell staining of sGRP78 in Ad/GRP78-infected MCF-7 cells. (B) Protein levels of sGRP78 as assessed by western blot. (C) Relative expression of sGRP78 in Ad/GRP78-infected MCF-7 cells is indicated as a fold change compared to control cells. (D) Effect of GRP78 overexpression on ER stress. (E) ER stress inducer tunicamycin stimulated sGRP78 expression. **p<0.01 vs Ad/β-gal-infected cells. M: membrane; C: cytosol; Tun: tunicamycin.

Considering that GRP78 is a master regulator involved in the regulation of ER stress and that ER stress is implicated in cancer survival, we next tested whether high sGRP78 expression is a consequence of ER stress resulting in GRP78 overexpression. As shown in Fig 3D, GRP78 overexpression did not change the phosphorylation status of PERK and IRE1α and expression of CHOP, indicating that ectopically expressed GRP78 did not induce ER stress. However, when MCF-7 cells were serum starved for 6 h, and then exposed to 2 μg/ml of the ER stress inducer tunicamycin for 24 h, sGRP78 expression was greatly increased in both Ad/β-gal- and Ad/GRP78-infected MCF-7 cells, suggesting that ER stress can upregulate the membrane distribution of GRP78.

**Fig 3:** Effect of sGRP78 on cell proliferation, apoptosis, and migration. (A) Effect of sGRP78 on cell proliferation. (B) Cell apoptosis with TUNEL. (C) Quantitative analysis of cell apoptosis. (D) Western blotting of key apoptosis-associated protein expression. (E) Images of MCF-7 cells in the wound-healing migration assay. (F) Quantitative analysis of wound closure in areas as marked in (E). (G) Mean values for the number of migrated MCF-7 cells counted in the areas as marked in (E). *p<0.05, **p<0.01. Ab: Anti-GRP78 antibody.

### Cell surface GRP78 positively regulates cell growth and migration

To characterize the possible association of sGRP78 with cell proliferation and migration, we used the goat polyclonal antibody raised against a peptide mapping at the N-terminus of GRP78 of human origin (anti-GRP78 antibody,N-20, Santa Cruz) to block the sGRP78 receptor function [25–28]. Ad/β-gal- and Ad/GRP78-infected MCF-7 cells were incubated in growth medium with 4 μg/ml anti-GRP78 antibody or normal goat IgG (Santa Cruz) for 24 h. The isotype-specific normal goat IgG was used as control. An MTT assay was carried out to determine cell proliferation. We found that GRP78 overexpression significantly increased cell proliferation and that GRP78-enhanced proliferation was mitigated by treatment with GRP78 antibody (Fig 3A). To induce cell apoptosis, serum-starved cells were treated with 25 ng/ml of TNFα for 24 h [29]. Cell apoptosis analysis by a TUNEL assay revealed that Ad/GRP78-infected cells were against TNFα-induced cell death, which is reversed by anti-GRP78 antibody (Fig 3B). Expression of cleaved caspase 3 and PARP, two key apoptosis regulatory proteins, supported that GRP78-suppressed apoptosis was deteriorated by anti-GRP78 antibody (Fig 3C). These data suggest that sGRP78 accelerates but neutralization of sGRP78 attenuates cell growth in MCF-7 cells.

RETRACTED

Next, we used a wound-healing assay to determine the impact of sGRP78 on cell migration. Monolayer MCF-7 cells were treated with 4 μg/ml of anti-GRP78 antibody or normal goat IgG at 48 h after infection with Ad/β-gal and Ad/GRP78. Photographs were taken immediately after wound induction and following 24 h incubation. As shown in Fig 3E–3G, we found that the wound healing abilities of GRP78-infected MCF-7 cells were markedly increased, compared with the control cells. In contrast, neutralization of sGRP78 by the anti-GRP78 antibody repressed wound healing capacity evidenced by decreased wound closure (Fig 3F) and number of migrated cells in the closed area (Fig 3G), suggesting that sGRP78 promotes cell migration.

### Cell surface GRP78 stimulates JAK2/STAT3 pathway

To figure out the relationship between sGRP78 and STAT3, we next investigated STAT3 phosphorylation in sGRP78 positive tumor tissues by western blot. We found that the tumor tissues with high expression of sGRP78 showed high levels of STAT3 phosphorylation (Fig 4A). Compared with adjacent non-tumor tissues, the cancer tissues show a ~2 fold increase of phosphorylated STAT3 (Fig 4B). A significant positive correlation was found with sGRP78 expression and STAT3 phosphorylation (r = 0.88, p<0.001; Fig 4C).

**Fig 4:** Stimulation of STAT3 phosphorylation by sGRP78. (A) Western blotting of sGRP78 protein and STAT3 phosphorylation in human breast tumor and non-tumor tissues. (B) Mean values of protein relative expression in (A). (C) Correlation of sGRP78 expression with STAT3 phosphorylation in human breast tumor. (D) STAT3 phosphorylation in Ad/GRP78-infected MCF-7 cells. (E) Quantitative analysis of STAT3 phosphorylation in (D). (F) Mitigation of sGRP78-induced STAT3 phosphorylation by treatment with anti-GRP78 antibody. *p<0.05, **p<0.01, ***p<0.001. N: non-tumor tissue; T: tumor tissue; M: membrane; C: cytosol; Ab: Anti-GRP78 antibody.

To address whether sGRP78 is responsible for increased STAT3 phosphorylation, MCF-7 cells were infected with Ad/β-gal and Ad/GRP78. The cells were harvested after 48 h of infection and protein phosphorylation was determined by western blot using specific antibody. We found that Ad/GRP78-infected cells showed enhanced phosphorylation of JAK2 and STAT3 (Fig 4D). Compared with Ad/β-gal infection, Ad/GRP78 infection resulted in ~3.4 fold increase of the ratio of p-STAT3 to STAT3 (Fig 4E). When Ad/GRP78-infected cells were administrated with 4 μg/ml of anti-GRP78 antibody for 24 h, the level of STAT3 phosphorylation dropped to basal line (Fig 4F and S1 Fig). These results indicate that sGRP78 activates JAK2/STAT3 pathway in MCF-7 cells.

RETRACTED

### STAT3 mediates cell surface GRP78-induced action

We then investigated the impacts of STAT3 on sGRP78-induced cell proliferation, apoptosis, and migration. To suppress STAT3 phosphorylation, Ad/β-gal- and Ad/GRP78-infected MCF-7 cells were incubated with 100 μM of a specific STAT3 inhibitor NSC74859 for 24 h or transduced with human STAT3/shRNA and control shRNA lentiviral particles for 48 h. We first observed that sGRP78-stimulated STAT3 phosphorylation could be suppressed by treatment with NSC74859 (S2 Fig) or by silencing of STAT3 (S3 Fig). Furthermore, NSC74859 treatment did not interfere with other signaling pathway (S2 Fig). Next, we used the same strategy to confirm the functional consequences of STAT3 inhibition on cell growth and migration. Cell proliferation, apoptosis, and migration were assessed by MTT, TUNEL, and wound healing assay, respectively. We found that the STAT3 inhibitor and STAT3/shRNA significantly attenuated cell proliferation (Fig 5A), increased apoptosis (Fig 5B), suppressed wound-closure (Fig 5C), and reduced the number of migrated cells (Fig 5D). Similarly, STAT3 knockdown significantly diminished effect of GRP78 overexpression on cell proliferation, apoptosis, and migration in MDA-MB-453 cells (S4 Fig). These data suggest that STAT3 might mediate sGRP78 function.

**Fig 5:** Effect of genetic and pharmacologic inhibition of STAT3 on cell proliferation, apoptosis, and migration in MCF-7 cells. (A) Inhibition of STAT3 on cell proliferation. (B) Inhibition of STAT3 on cell apoptosis. (C) Inhibition of STAT3 on wound closure. (D) Inhibition of STAT3 on the number of migrated. *p<0.05, **p<0.01, ***p<0.001, NSC: NSC74859, a specific STAT3 inhibitor.

## Discussion

Recent studies have established the critical roles of sGRP78 in the pathogenesis of cancer growth, metastasis, and resistance to chemotherapy [9, 10, 15, 16]. In this study, we show that sGRP78 is a novel regulator in modulating cell growth and metastasis in breast cancer cells. Importantly, we confirm that sGRP78-induced activation of STAT3 is a key event in breast cancer cell proliferation and migration.

In agreement with early studies showing that GRP78 relocates to the cell membrane in malignant but not in benign cells [8], we found that sGRP78 was highly expressed in human breast tumor, compared with adjacent non-tumor tissues (Fig 1A–1C). In addition, our data demonstrates that the levels of sGRP78 were positively associated with pathological stage of breast cancer (Fig 1D and Table 1), suggesting that sGRP78 might contribute to breast cancer progression. This view is supported by our *in vitro* studies. Human MCF-7 breast cancer cells have the weakest invasive potential [30] and dormant characteristics [31], as well as the lowest endogenous levels of GRP78 protein expression in the cancer cell lines tested [24]. Our results found that overexpression of GRP78 in MCF-7 cells result in high-level expression and membrane distribution of GRP78 (Fig 2A–2C), accompanied by significantly increased cell proliferation, reduced cell apoptosis, and accelerated cell migration (Fig 3). This important impact of sGRP78 on the promotion of cancer cell growth and migration was further confirmed by using a specific antibody to inhibit sGRP78 function. Our results showed that immunoneutralization of sGRP78 attenuated the Ad/GRP78-induced impact on cell growth and migration (Fig 3), suggesting that sGRP78 is responsible for cancer cell growth and migration. Taken together, our findings strongly indicate that sGRP78 contributes to breast cancer survival and migration.

RETRACTED

It has been reported that binding of N- and C-terminal anti-GRP78 antibodies (N-20 and C-20) generates distinct impacts on GRP78 signaling. The carboxyl terminal GRP78 antibodies (C-20) inhibit GRP78 signaling, while amino terminal GRP78 antibodies (N-20) stimulate GRP78 signaling [16, 32]. In contrast, some studies have demonstrated that anti-GRP78 N-20 antibody can block sGRP78 functions effectively in many human cancers [25–28]. Our preliminary studies showed that either N-20 or C-20 antibody could impede sGRP78 signaling towards cell proliferation and migration (Data not shown). However, we do not understand the underlying mechanism. The further work is necessary to decipher why antibodies directed against these different GRP78 epitopes both impact STAT3 signaling.

It is well known that GRP78 plays a key role in the regulation and induction of ER stress [11, 33], which has a profound effect on cancer cell proliferation and survival [33, 34]. The question is whether sGRP78 stimulates cell growth and migration by ER stress. Our results found that the ER stress inductor tunicamycin dramatically increased the level of sGRP78 in MCF-7 cells (Fig 2E), consistent with previous observations that have demonstrated cell surface localization of GRP78 may be induced by thapsigargin in normal or cancer cells, including MCF-7 cells [35, 36]. However, overexpression of GRP78 did not lead to ER stress or an unfolded protein response (UPR) (Fig 3D), suggesting that sGRP78 function is independent from ER stress.

RETRACTED

STAT3 has been demonstrated to contribute to tumor growth through regulating protein expression of other signaling molecules, apoptosis, and the cell cycle [37]. In the present study, we found a positive correlation existed between sGRP78 levels and STAT3 phosphorylation in human breast cancer tissues (Fig 4A–4C). The elevated phosphorylation of STAT3 and its upstream kinases JAK2 was also expressed in Ad/GRP78-infected MCF-7 cells (Fig 4D and 4E). Inhibition of sGRP78 functions by GRP78 antibody mitigated Ad/GRP78-induced STAT3 phosphorylation. These findings indicate that sGRP78 can activate the JAK2/STAT3 pathway. In addition, genetic and pharmacological inhibition of STAT3 significantly attenuated Ad/GRP78-induced cell growth and migration (Fig 5 and S4 Fig). Thus, our findings are intended to support a conclusion that STAT3 mediates sGRP78 action on breast cancer cell proliferation and migration.

sGRP78 functions as a receptor on the cell surface [38]. Through forming complexes with specific cell surface proteins, sGRP78 regulates signal transduction of cancer cells, such as the α2-macroglobulin-induced signal [39], TGF-β signaling [40, 41], Ras/MAPK and PI3K/AKT signal pathways [9, 10, 15], Smad2/3 pathways [27], and the mTORC1 and mTORC2 signaling pathways [42], leading to cancer growth and metastasis. In this study, we found that anti-GRP78 antibodies did not co-immunoprecipitate with STAT3 and JAK2 in whole cell lysates of sGRP78 positive tumor tissues and Ad/GRP78-infected MCF-7. Conversely, an anti-STAT3 antibody also did not cross-immunoprecipitate with GRP78 (data not shown), consistent with the previous study showing that STAT3 is not associated with GRP78 [43]. These results suggest that sGRP78 modulates the STAT3 pathway by an indirect manner.

The PI3K and STAT3 signaling pathways were historically regarded as two distinct regulatory networks but emerging evidence suggests that the two pathways actually interact with each other and their interplay may be critical to promote tumor growth [44]. In some human tumor cell lines, the enhanced phosphorylation of STAT3 is inhibited by the PI3K inhibitor [45]. On the contrary, pretreatment with the JAK2/STAT3 pathway inhibitor AG490 or stattic inhibited propofol-induced AKT phosphorylation [5, 46], suggesting that the link between PI3K and STAT3 pathways is significant in human cancers. Given that the dual activation and crosstalk of cytoprotective PI3K/AKT and JAK2/STAT3 pathways exists in sGRP78 positive cancer cells, it is possible that sGRP78-stimulated PI3K/AKT signaling is involved in the regulation of STAT3 phosphorylation. More studies are needed to further define this possibility.

RETRACTED

In summary, our results demonstrate, for the first time, that sGRP78-dependent STAT3 activation increases breast cancer cell growth and migration. This finding might further lead to the development of new therapeutic approaches targeted against breast cancer with high level of sGRP78.

## Supporting Information

S1 Fig Overexpression of GRP78 in MDA-MB-453 cells. MDA-MB-453 cells were infected with Ad/GRP78 or Ad/β-gal in serum free medium for 4 h, and then incubated in growth medium. Forty-eight hours late after infection, the cells were cultured in the present or absent of 4 μg/ml anti-GRP78 antibody or isotype-specific serum for 24 h. Membrane fraction was isolated as described in Material and Methods. Western blot was performed to detect protein expression and its phosphorylation by using specific antibodies. (A) Protein levels of sGRP78 as assessed by western blot. (B) Effect of GRP78 neutralization by anti-GRP787 antibody on JAK2/STAT3 pathway. Ab: anti-GRP78 antibody.
(TIF)

S2 Fig NSC74859 suppressed GRP78-stimulated STAT3 phosphorylation in Ad/GRP78-infected MCF-7 cells. MCF-7 cells were infected with Ad/GRP78 or Ad/β-gal in serum free medium for 4 h, and then incubated in growth medium. Forty-eight hours late after infection, MCF-7 cells were treated with 100 μM of specific STAT3 inhibitor NSC74859 for 2 h [47, 48]. Western blot was performed to detect STAT3 protein expression and its phosphorylation by using specific antibodies. (A) Representative western blot image of STAT3 phosphorylation. (B) Quantification of phosphorylated STAT3 in (A). (C) Representative western blot image of irrelevant signaling molecules. *p<0.05 vs Ad/β-gal control, ##p<0.01 vs Ad/GRP78 group.
(TIF)

S3 Fig STAT3/shRNA lentiviral particles mitigated STAT3 expression and abolished STAT3 phosphorylation. MCF-7 cells were infected with human STAT3/shRNA and control shRNA lentiviral particles at 48 h after Ad/GRP78 or Ad/β-gal (as controls) infection. 48 hours later, the cells were harvested and western blot was performed to detect STAT3 protein expression and its phosphorylation by using specific antibodies.
(TIF)

S4 Fig Effect of STAT3 knockdown on cell proliferation, apoptosis, and migration. Ad/β-gal- and Ad/GRP78-infected MDA-MB-453 cells were transduced with human STAT3/shRNA and control shRNA lentiviral particles for 48 h. Cell proliferation, apoptosis, and migration were assessed by MTT, TUNEL, and wound healing assay, respectively. (A) STAT3 knockdown on cell proliferation. (B) STAT3 knockdown on cell apoptosis. (C) STAT3 knockdown on wound closure. (D) STAT3 knockdown on the number of migrated MDA-MB-453 cells. *p < 0.05 vs Ad/β-gal- and STAT3/Scrambled-infected cells; #p < 0.05 vs GRP78-overexpressed and STAT3/Scrambled-infected cells.
(TIF)
